The article "Tropheryma whipplei: A Common Bacterium in Rural Senegal" was retracted in 2025. Reasons: lack of ethics approval or compliance; a conflict of interest; concerns about the welfare of human subjects.

# *Tropheryma whipplei*: A Common Bacterium in Rural Senegal

**DOI:** 10.1371/journal.pntd.0001403

**Published:** 2011-12-20

**Authors:** Alpha Kabinet Keita, Hubert Bassene, Adama Tall, Cheikh Sokhna, Pavel Ratmanov, Jean-François Trape, Didier Raoult, Florence Fenollar

**Affiliations:** 1 Unité de Recherche sur les Maladies Infectieuses et Tropicales Emergentes, URMITE CNRS-IRD 198 UMR 6236, Université de la Méditerranée, Faculté de Médecine, Marseille, France; 2 Unité de Recherche sur les Maladies Infectieuses et Tropicales Emergentes, URMITE CNRS-IRD 198 UMR 6236, Institut de Recherche pour le Développement (IRD), Campus commun UCAD-IRD of Hann, BP 1386, CP 18524, Dakar, Senegal; 3 Unité d'Epidémiologie, BP 220, Institut Pasteur de Dakar, Dakar, Senegal; 4 Department of Public Health and Health Services Management, Far Eastern State Medical University, Khabarovsk, Russia; University of Washington, United States of America

## Abstract

**Background:**

*Tropheryma whipplei* is known as the cause of Whipple's disease, but it is also an emerging pathogen, detected in stool, that causes various chronic localized infections without histological digestive involvement and is associated with acute infections, including gastroenteritis and bacteremia.

**Methods/Principal Findings:**

We conducted a study in 2008 and 2009 using 497 non-diarrheic and diarrheic stool samples, 370 saliva samples, 454 sera samples and 105 samples obtained from water samples in two rural Sine-Saloum villages (Dielmo and Ndiop) in Senegal. The presence of *T. whipplei* was investigated by using specific quantitative PCR. Genotyping was performed on positive samples. A serological analysis by western blotting was performed to determine the seroprevalence and to detect seroconversion. Overall, *T. whipplei* was identified in 31.2% of the stool samples (139/446) and 3.5% of the saliva samples (13/370) obtained from healthy subjects. The carriage in the stool specimens was significantly (*p*<10^−3^) higher in children who were between 0 and 4 years old (60/80, 75%) compared to samples obtained from individuals who were between 5 to 10 years old (36/119, 30.2%) or between 11 and 99 years old (43/247, 17.4%). The carriage in the stool was also significantly more common (*p* = 0.015) in subjects with diarrhea (25/51, 49%). We identified 22 genotypes, 16 of which were new. Only one genotype (#53) was common to both villages. Among the specific genotypes, one (#52) was epidemic in Dielmo (15/28, 53.4%, *p*<10^−3^) and another (#49) in Ndiop (27.6%, *p* = 0.002). The overall seroprevalence was estimated at 72.8% (291/400). Seroconversion was detected in 66.7% (18/27) of children for whom PCR became positive in stools between 2008 and 2009.

**Conclusions/Significance:**

*T. whipplei* is a common bacterium in the Sine-Saloum area of rural Senegal that is contracted early in childhood. Epidemic genotypes suggest a human transmission of the bacterium.

## Author Summary

*Tropheryma whipplei* is known as the cause of Whipple's disease. It is also an emerging pathogen, detected in stool that causes various chronic localized infections without histological digestive involvement and is associated with acute infections, including gastroenteritis and bacteremia. We have studied the presence of *T. whipplei* on non-diarrheic and diarrheic stool samples, saliva samples, and sera samples in two rural Sine-Saloum villages (Dielmo and Ndiop) in Senegal. *T. whipplei* was identified in 31.2% of the stool samples and 3.5% of the saliva samples from healthy subjects. The carriage in the stool specimens was higher in children who were between 0 and 4 years old (75%) compared to samples obtained from individuals between 5 to 10 (30.2%) or between 11 and 99 (17.4%). The carriage in the stool was also more common in subjects with diarrhea (49%). We identified 22 different genotypes of *T. whipplei*. Only one genotype was common to both villages. Among the specific genotypes, one was epidemic in Dielmo and another in Ndiop. The seroprevalence was estimated at 72.8%. *T. whipplei* is a common bacterium in the Sine-Saloum area of rural Senegal that is contracted early in childhood. Epidemic genotypes suggest a human transmission of the bacterium.

## Introduction

Traditionally, *Tropheryma whipplei* was considered to be a rare bacterium that typically caused the classic form of Whipple's disease, which is characterized by histologically periodic acid-Schiff–stained bacilli in infected small-bowel macrophages [1]–[3]. However, this well-known pathology, described primarily in Caucasian men and very seldomly in people of African origin, represents only one rare clinical manifestation of *T. whipplei* infection [2], [4], [5]. Recent studies have shown that a wide spectrum of infections is caused by *T. whipplei* [2], [5]–[9]. The bacterium also causes localized chronic infections without histological digestive involvement, such as endocarditis, spondylodiscitis, meningoencephalitis, uveitis, and pneumonia [2], [5]–[9]. In addition, *T. whipplei* DNA was recently found to be highly prevalent (15%) in stool samples obtained from 241 children who were between 2 to 4 years old in France and had gastroenteritis, but it was not detected in a control group of children of the same age without gastroenteritis [10]. *T. whipplei* DNA has also been detected in stool and saliva specimens obtained from healthy individuals, and its prevalence depends primarily on geographic area [11]–[13]. In Europe, the prevalence of this bacterium in stool samples is estimated to be between 1% and 11% among the healthy general population and between 12% and 26% among sewage workers [14]–[16]. In France, the carrier prevalence of *T. whipplei* in saliva is estimated to be 0.2% in the general population and 2.2% among sewage workers [14], [15]. In a preliminary study of 150 healthy children conducted in 2 villages in Senegal (Dielmo and Ndiop), the prevalence of *T. whipplei* in stool samples was 30% for children between eight months and two years old and 44% in children between two and ten years old [17]. More recently, a study using 204 blood samples obtained from febrile patients who were negative for malaria in these same villages found *T. whipplei* DNA in 13 samples (6.4%) [17]. Here, we have extended this research to the entire population of these 2 villages to confirm these preliminary results and establish the kinetics of *T. whipplei* carriage in stools from April 2008 to April 2009. We also extended the study to include saliva samples from healthy individuals, stool samples from diarrheal patients and additional water samples.

## Materials and Methods

### Ethics statement and the populations of the two villages

This cohort study was approved by the national ethics committee of Senegal and the local ethics committee of IFR 48 (agreement number 09–022, Marseille, France). Written informed consent was obtained from all individuals, including patients and parents or legal guardians of all children.

From April to October 2009, we performed studies among the populations of Dielmo (13°43′N, 16°25W) and Ndiop (14° 33′ N, 16°15′ W), which are two villages in the Sine-Saloum region of Senegal. These villages are included in the Dielmo project, a longitudinal prospective study initiated in 1990 for the long-term investigation of host–parasite associations [18], [19].

In April 2009, at the time of the samplings of saliva and stools specimens, the population of Dielmo was composed of 379 people (200 females), including 63 children (17%) of less than 5 years of age and the population of Ndiop was composed of 274 (154 females), including 55 children of less than 5 years of age (20%).

### Human samples

#### Stool and saliva samples

In April 2009, 446 stool and 370 saliva samples from healthy individuals were analyzed. In addition, 51 stool samples, from July to October 2009, from patients who developed diarrhea, defined by the presence of at least 3 stools per day, were also tested. After collection, the stool and saliva specimens were mixed with 2.5 or 1 ml absolute ethanol, respectively, for storage and transportation at room temperature to our center in France.

#### Sera

As a part of the Dielmo project, capillary sampling was conducted monthly among all of the individuals included in the study. The current analysis focused on samples obtained in June and July 2008 for the seroprevalence study (400 sera). For the seroconversion study, our analysis involved 27 people; two serum samples were obtained from each person (the first collected on May 2008 and the second collected on May 2009). Sera were stored at −20°C and transported to our laboratory in an ice box.

### Environmental samples

A total of 105 samples, including 6 samples obtained from wells (145 ml of water from each one), 92 samples obtained from canaris (vases used to store water; 50 ml of water from each one), and 7 samples from opens water sources in the region (rivers and marshes; 200 ml of water from each one) were analyzed. These samples were stored at room temperature for transport to our laboratory in France. On arrival, the water samples were filtered through a 0.22 µm membrane (Millipore). The membrane was then immersed in 2 ml of PAS buffer (Page's Amoeba Saline, Unipath Ltd.Wade Road, UK), and the supernatant was stored at −80°C until analysis.

### Molecular assays

Approximately one gram of stool, 200 µl of saliva and 200 µl of water were individually submitted for DNA extraction using a BioRobot MDx workstation (QIAGEN, Valencia, CA, USA) according to the manufacturer's recommendations and protocols. Quantitative real-time PCR (qPCR) targeting repeated sequences (repeat-PCR) was performed using a LightCycler® instrument (Roche Diagnostics, Meylan, France) with a QuantiTect Probe PCR Kit as described previously [15], [20]. First, specimens were tested using the Twhi3F (5′-TTGTGTATTTGGTATTAGATGAAACAG-3′) and Twhi3R (5′-CCCTACAATATGAAACAGCCTTTG-3′) primer pair and the specific TaqMan probe Twhi3 (6-FAM-GGGATAGAGCAGGAGGTGTCTGTCTGG-TAMRA). When the specimen was found to be positive using this assay, the result was confirmed through a second round of qPCR analysis using the Twhi2F (5′-TGAGGATGTATCTGTGTATGGGACA-3′) and Twhi2R (5′-TCCTGTTACAAGCAGTACAAAACAAA-3′) primer set and the Twhi2 probe (6-FAM-GAGAGATGGGGTGCAGGACAGGG-TAMRA). To validate the test, we used positive and negative controls as previously reported [15], [20].

Genotyping of *T. whipplei* was performed as described previously [21]. Each of the four highly variable genomic sequences (HVGSs) obtained from each specimen were compared with those available in both the GenBank database and our internal laboratory database to determine their corresponding genotype. When a new sequence was obtained, we have systematically performed two additional rounds of sequencing to confirm it. The sensitivity levels of repeat-PCR and PCR assays used for genotyping were evaluated on DNA extracted from 10-fold dilutions of a suspension of 10^4^ *T. whipplei* strain Marseille-Twist (ATCC VR-1528) bacterium.

Finally, as we have not previously amplified *T. whipplei* in water, we have checked the feasibility to amplify it from water artificially infected. Thus, we have infected 5 flasks of 50 ml of sterile water with 10-fold dilutions of a suspension of 10^4^ *T. whipplei*. The water samples were then filtered and submitted to DNA extraction and repeat-PCR as reported above.

### Western blot assays

Serological assays were performed by western blot. Native and deglyclosylated samples obtained from total bacterial extracts were prepared for SDS-PAGE as previously reported [22]. Proteins were separated by SDS-PAGE and transferred onto nitrocellulose membranes. The protein concentration of the samples was determined using a Biorad reagent (Hercules, CA, USA). The membranes were immersed in PBS supplemented with 0.2% Tween 20 and 5% non-fat dry milk (blocking buffer) for 1 h at room temperature before incubation with primary sera (diluted 1∶1,000 in blocking buffer) for 1 h at room temperature. The membranes were then washed three times with PBS-Tween 20, and immunoreactive spots were detected by incubating the membranes for 1 h at room temperature with a peroxidase-conjugated goat anti-human antibody (Southern Biotech, Birmingham, AL, USA) diluted 1∶1,000 in the blocking buffer. Detection was performed using chemiluminescence (Enhanced Chemiluminescence Western Blotting Analysis System; Amersham Biosciences, Uppsala, Sweden) with an automated film processor (Hyperprocessor; GE Healthcare).

### Statistical analysis

Data were analyzed using PASW statistics 17 software (SPSS, Chicago, IL, USA). Non-parametric values were compared using the chi-square test. Statistical significance was defined as p<0.05. The corrected chi-squared test or the Fisher's exact test was used where indicated.

## Results

### Analysis of stool and saliva specimens from healthy people and environmental sources

In this study, stool samples from 446 individuals aged from 1 month to 87 years old (mean age 20±18.71 years) were collected in April 2009. Among these samples, 139 (31.2%, 95% confidence interval [CI] 26.9%–35.6%) presented a positive PCR in Dielmo and Ndiop. Sixty-two out of 219 tested in Dielmo (28.3%) were positive, compared to 77 out of 227 in Ndiop (33.9%, p = 0.2). *T. whipplei* carriage in stools was higher in children aged from 0 to 4 years (60 out of 80, 75%, Figure 1). The prevalence in this age group was significantly different from other age groups (p<10^−3^; 60/80 versus 36/119 for the group from 5 to 10 years old and 43/247 for the group from 11 to 87 years old). Saliva samples were collected from 370 people aged from 4 to 91 years (mean age 27±19.5 years). *T. whipplei* carriage was found to be 3.5% (13/370, 95% CI 1.9%–5.8%, Figure 2) in these samples, and the prevalence in Ndiop (5.9%, 12/201) was significantly different from that detected in Dielmo 0.6% (1/169, p = 0.005). *T. whipplei* carriage in saliva was higher in the 5 to 10 years old age group (8 out of 83, 9.6%, p = 0.02). Among the 150 children tested in 2008, stool samples were obtained from 118 in 2009. Of 118, 52 (44.1%) were negative over the two-year period. A total of 30 of 118 (25.4%) were positive in April 2008 and 2009. Twenty-eight children whose stools were negative in April 2008 were determined to be positive in April 2009 (23.7%). Stool and saliva samples were available for 294 persons in April 2009. Of these sample sets, 219 were negative in both stool and saliva (74.5%); 62 (21.1%) were positive in stool but negative in saliva, 13 were positive in both samples (4.4%) and none was positive in saliva and negative in stools. The villages of Dielmo and Ndiop contain 82 households. In this study, we analyzed samples obtained from individuals residing in 58 different households. In 52 of the households, none of the residents presented *T. whipplei* DNA in their saliva samples; among these individuals, 126 of 431 (29.2%) were positive for *T. whipplei* in stool specimens. In the 6 remaining households, at least one of the residents presented *T. whipplei* DNA in their saliva sample; among those living in these households, 48 of 147 (32%) were positive for *T. whipplei* in stool specimens. Finally, *T. whipplei* DNA was not detected in the 105 water samples tested even if we were able to amplify *T. whipplei* among all the flasks artificially infected.

**Figure 1:** Prevalence of *T. whipplei* in stool samples from healthy individuals in Dielmo and Ndiop.

**Figure 2:** Prevalence of *T. whipplei* in saliva samples from healthy individuals in Dielmo and Ndiop.

### Analysis of stools from diarrheic patients

Fifty-one diarrheal stool samples (Figure 3) were analyzed during our study (mean age 4±3.2 years). *T. whipplei* was detected in 10 of 20 samples in Dielmo (50%) and 15 of 31 samples in Ndiop (48.4%). The prevalence of *T. whipplei* in patients with diarrhea, 49% (25/51, 95% CI 35.2%–62.6%), was significantly higher (p = 0.015) than that found among controls (139/446, 31.2%). When we analyzed our data according to age, our primary observation was that *T. whipplei* DNA was never detected in diarrheic patients who were more than 11 years old, whereas it was detected in half of the patients under 11 years old.

**Figure 3:** Prevalence of *T. whipplei* in stool samples from diarrheic individuals in Dielmo and Ndiop.

### Genotyping

Genotyping data were available when high DNA loads were found, which occurred in 61 specimens (53 stool and 8 saliva samples) from 57 people (28 in Dielmo and 29 in Ndiop, Figure 4 and Table S1). Indeed, in comparisons of the detection capacities of the molecular assays, we were able to detect 1 DNA copy of standard control DNA when our repeat-PCR was used and only 10 copies when our PCR assays for genotyping were used. The additional rounds of sequencing have allowed to obtain the same sequence each time confirming the robustness of our data. All the nucleotide sequences detected in this study have been deposited in GenBank and their reference numbers are presented in Table S2. Overall, 22 different genotypes were detected, including 16 new genotypes (genotypes 63–81); all of these were specific to Senegal. Only one genotype (#53) was common to the two villages, although it was identified more frequently in Ndiop (7/9, 77.8%) than in Dielmo (2/9, 22.2%; p = 0.1). Otherwise, 26 of 28 individuals from Dielmo (93%) and 22 of 29 from Ndiop (76%) were infected with genotypes specific to each village (Figures 5 and 6). Genotype 52 was observed specifically in 15 of 28 individuals tested in Dielmo (53.4% versus 0 in Ndiop, p<10^−3^). Genotype 49 was present exclusively in 8 of the 29 individuals tested in Ndiop (27.6% versus 0 in Dielmo, p = 0.002). For 4 people out of 57, a genotype was obtained for both saliva and stools specimens. The same genotype was identified in both samples for the 4 individuals.

**Figure 4:** Phylogenetic diversity of 81 genotypes of *T. whipplei* obtained from 151 samples. The phylogenetic tree is constructed using the UPGMA method. Sequences from the four HVGs were concatenated. The HVGs 1, 2, 3, and 4 have intervened respectively in 24, 22, 27 and 18 different combinations. Opposite the genotype, the places in which the genotype has been detected are presented with between the parentheses the number of different samples in which the genotype has been detected. All the 57 genotypes detected in stool and saliva specimens during our study in Dielmo and Ndiop (Senegal) are highlighted in grey.

**Figure 5:** Data about *T. whipplei* according to the localization of the households in Dielmo. The prevalence of *T. whipplei* in stool specimens and seroprevalence are presented. The genotypes are indicated when they were identified at least two times in the village. The map in this image is © 2011 Google and is not subject to the terms of the Creative Commons Attribution License of the rest of the manuscript.

**Figure 6:** Data about *T. whipplei* according to the localization of the households in Ndiop. The prevalence of *T. whipplei* in stool specimens and seroprevalence are presented. The genotypes are indicated when they were identified at least two times in the village. Genotypes 48, 75, and 81 were specific to individual households. The map in this image is © 2011 Google and is not subject to the terms of the Creative Commons Attribution License of the rest of the manuscript.

### Serology

#### Seroprevalence study

Serological analysis was performed on 400 sera samples obtained from healthy people who were between 3 and 78 years old (mean age 20.5±13.4). Among them, 291 (72.8%, 95% CI 68.2%–76.9%, Figures 5, 6 and 7) exhibited a serological response directed against *T. whipplei*. The seroprevalence was 69.5% (139/200) in Dielmo and 76% (152/200) in Ndiop (p = 0.178). The highest seroprevalence (68 out of 86, 79.1%) was observed among children who were between 5 and 10 years old versus seroprevalences of 222/312 (71.2%, p = 0.18) and 1/2 (p = 0.38) among individuals who were between 10 and 78 years old and 0 and 4 years old, respectively.

**Figure 7:** Seroprevalence of *T. whipplei* in Dielmo and Ndiop.

#### Seroconversion study

The stool samples from 27 children who were between 5 months and 10 years old (mean age 3.8 years ±2.2) were negative for *T. whipplei* DNA in 2008 but positive in 2009. Among these individuals, 18 presented a seroconversion for *T. whipplei* (66.7%, 95% CI 47.6%–82.4%). Eight (29.6%) exhibited a positive serology in both 2008 and 2009. An eight-month-old baby showed no serological reaction after these two years. Thus, the children for whom PCR became positive for *T. whipplei* from 2008 and 2009 had significantly developed a seroconversion for *T. whipplei* (18/27 versus 8/27 and 1/27, p<10^−3^).

### Concordance between the presence of *T. whipplei* in stool and serological responses

A concordance study was conducted between the presence of *T. whipplei* in stool among children younger than 11 years old and the presence of an immune response against *T. whipplei* as determined by western blot analysis. We identified a link between the presence of *T. whipplei* in the stool and the presence of an immune response against the bacterium. Among the ≤6-years old age group, no patients who presented negative PCR results exhibited a serological response (Table 1). However, in the 5- to 10-year-old age group, 7 children who presented negative stool-sample PCR results exhibited an immune response against *T. whipplei*.

**Table 1:** Concordance between the presence of *T. whipplei* in stool specimens and serological responses for children.

		*T. whipplei* DNA in stools samples		
		Presence	Absence	Total
		Data for 8 children younger than 6 years old.		
***T. whipplei*** ** antibodies**	**Presence**	4	0	4
	**Absence**	1	3	4
	**Total**	5	3	8

		Data for 10 children aged from 6 to 10 years old		
***T. whipplei*** ** antibodies**	**Presence**	9	7	16
	**Absence**	1	3	4
	**Total**	10	10	20

## Discussion

The validity of the reported data is based on strict experimental procedures and controls, including positive and negative controls used to validate the test. Each positive PCR result was confirmed with the successful amplification of an additional DNA sequence, and all sequences with at least one mutation were systematically confirmed through 2 additional rounds of sequencing. Therefore, we are confident in the results presented here: *T. whipplei* is endemic. Although twenty-two different genotypes that are specific to Senegal have been detected, confirming the genetic heterogeneity of *T. whipplei* [10], [13], [21], only genotype 53 was common to both villages. This genotype was epidemic in Ndiop, where it affected 24% of the positive individuals [13]. All of the other detected genotypes were specific to each village and were endemic. Among them, one genotype (#49) was detected in 27.6% of the affected individuals in Ndiop and another (#52) was detected in 53.6% of the affected individuals in Dielmo. Thus, the fact that almost half of the people were affected by the same genotype cannot be attributed to chance. This important circulation of specific genotypes confirms the theory that *T. whipplei* is contagious. One of our initial hypotheses was that the water, mainly the stored water for drinking represented a possible source of contamination for the population; however, our results allowed us to refute this hypothesis [13]. The lack of detection of *T. whipplei* in our environmental samples may be explained by the fact that toilets in each household are constructed by the principle of septic tank, so the excrements are not allowed to be freely distributed all over. Villagers used as a drinking water relatively deep (>20 m) covered wells only, so the contact of the drinking water with the excrements is minimized. Besides, the fact that *T. whipplei* is a fastidious bacterium, suggests that it cannot propagate in water. Thus, even if minuscule quantities of bacterium may invade water with human excrements, they are, probably, below the threshold of identification and do not play important epidemiological role. Moreover, environmental sources do not explain the circulation in the two villages. Our hypothesis is that the bacterium can be transmitted through saliva [23].

In France, *T. whipplei* has recently been identified as an agent of gastroenteritis in young children, either alone or in combination with other pathogens [10]. In parallel, an in *vivo* model of infection with *T. whipplei* in mice was developed that further confirmed the role of *T. whipplei* as an agent of gastroenteritis [24]. In our study, the analysis of children who were between 5 and 10 years old confirms a link between *T. whipplei* and gastroenteritis, although the interpretation of the results from the 4-year-old and younger group is more difficult. The high prevalence of carriage of *T. whipplei* in young subjects, the small number of diarrheal stool samples analyzed and the occurrence of very early primary infections are factors that limit the interpretation of our data. Nevertheless, it is important to emphasize that the spectrum of the manifestations of primary infection due to *T. whipplei* seems to be variable and includes gastroenteritis, pneumonia and bacteremia [10], [17], [25], [26]. Furthermore, patients may also develop multiple infections, including diarrhea or successive infections. It will be necessary to design a specific study in order to better determine the prevalence of *T. whipplei* among young children with diarrhea in rural Senegal as well as those of other defined pathogens and to evaluate the percentage of co-infection.

The prevalence of *T. whipplei* in stool specimens obtained from children under 5 years of age is 75%, a percentage that decreases among the 5 to 10-year-old age group (30%). The prevalence in individuals older than 10 years old (17.4%) is lower than that in children under 10 years old, although it is higher than that observed among the general population of Europe [14], [15]. A discrepant prevalence of *T. whipplei* in saliva is observed between the 2 villages. Discrepancies between these 2 villages have been previously observed regarding the incidence of several infectious diseases such as flea-borne spotted fever, tick-borne relapsing fever, malaria, and Q fever that are more prevalent in Dielmo than in Ndiop [27]. However, reasons for the significantly different prevalence of these infectious diseases in the 2 geographically close villages remain unexplained until now. In our study, a higher prevalence of *T. whipplei* carriage in saliva is observed in Ndiop in comparison to Dielmo. We have no explanation for this. One hypothesis may be a different lifestyle between the 2 populations, with closer contacts between people in Ndiop in comparison to Dielmo but this suggestion as well as other hypotheses should be studied.

This is the first study on the seroprevalence of *T. whipplei* performed in Africa using a recently described methodology [22]. This western blot-based approach revealed that subjects in France who were healthy carriers of *T. whipplei* exhibited a more intense immune response compared to those with classic Whipple's disease [22]. In our study, one of the 2 children under 5 years old tested positive. For the children between 5 and 10 years old, the seroprevalence is 79%, and it is 71.2% for people older than 10 years old. These data suggest that almost two thirds of the population in the Sine-Saloum area of rural Senegal have been infected with *T. whipplei*, confirming that this bacterium is common. Very few sera from very young children have been tested. However, notably for children younger than 6 years old, the presence of a serological response was systematically associated with the presence of *T. whipplei* DNA in stool specimens, whereas for children between 5 and 10 years old, almost half who presented a serological response did not present *T. whipplei* DNA in their stool specimens. This suggests a primary infection that occurs before individuals are 5 years old and a later elimination of the bacterium. Taken together, these seroprevalence and seroconversion data, in addition to the high prevalence of *T. whipplei* in stool samples from young children, are strong arguments supporting the idea of primary infections occurring in young children. Finally, there is also a network of circulation of epidemic genotypes between households in each village, as well as the 3 epidemic genotypes that are specific for 2 households in Ndiop.

Overall, *T. whipplei* is an emerging pathogen since the first culture of the bacterium 10 years-ago has allowed the development of efficient molecular tools leading to its more common detection. The first data have been obtained in France with approximately 2% of positive in stools from the general population but more impressive are the data observed in this area of rural Senegal with 31.2% of positivity in stools. The high incidence of *T. whipplei* in rural Senegal and the increasing spectrum of clinical manifestations due to the bacterium allow us to suggest that *T. whipplei* infection might be a major public health concern in West Africa. The existence of epidemic genotypes and its absence from environmental samplings suggests a human transmission of the bacterium. We speculate that *T. whipplei* is a contagious bacterium that is contracted early in childhood and is responsible for an underestimated number of acute clinical manifestations. Only a small number of individuals with specific immune deficiencies, which have not yet been determined, will develop classic Whipple's disease or other chronic localized infections. Further studies in Senegal will help us to elucidate the natural history of *T. whipplei*.

## Supporting Information

Checklist S1 **STROBE checklist.**
(DOC)

Table S1 **List of genotypes detected in the 2 villages (A) and in the households (B) studied.**
(DOC)

Table S2 **Reference numbers of the nucleotide sequences detected in this study and deposited in GenBank.**
(DOC)
